The article "Design of Personalized Ideological and Political Education Resource Recommendation System in the Online Education Platform in the Network Environment" was retracted in 2023. Reasons: signs of a paper mill; suspected computer-generated content; unreliable results or conclusions; concerns about the data.

# Design of Personalized Ideological and Political Education Resource Recommendation System in the Online Education Platform in the Network Environment

**DOI:** 10.1155/2022/3845749

**Published:** 2022-07-13

**Authors:** Tao Yang, Zhiqun Duan

**Affiliations:** ^1^Department of Automotive Engineering, Hebei Vocational University of Industry and Technology, Shijiazhuang 050091, Hebei, China; ^2^Department of Intelligent Manufacturing, Hebei Vocational University of Industry and Technology, Shijiazhuang 050091, Hebei, China

## Abstract

In the network environment, online ideological and political education is facing many challenges, the mainstream values of education have been impacted, and the backward educational model, single communication method, and solidified educational content are not conducive to the smooth progress of ideological and political education. However, at the same time, its innovation also ushers in development opportunities, rich educational resources, information platforms, diversified education subjects, strongly targeted education models, etc., which can become favorable factors for educational innovation. To this end, online educators should seize the development opportunities, grasp the good network environment, actively build a network platform for ideological and political education, create a personalized ideological and political education resource recommendation system, and reform the ideological and political education classroom, effectively playing the role of the main position of educating people. Online education breaks through the limitations of time and space, allowing students to get guidance from online teachers without leaving home, and is favored by more and more primary and secondary school students because of its unique advantages. At present, the forms of tutoring for off-campus online education in China are diverse, and there are several specific teaching modes. Whether online teaching can meet the needs of users is a problem worth studying.

## 1. Introduction

In recent years, with the development of Internet technology, online education has also come into being, and online education has been favored by more and more users because of its convenience, intelligence, and many other advantages. Relying on intelligent detection tools to assist teaching, online education can provide “personalized” tutoring to solve the learning problems of different user groups; with the popularity of 5G, the problem of network latency will be solved, and teachers and students will communicate more smoothly through the Internet. In recent years, a series of favorable policies and social events have promoted the steady and rapid development of online education.

In February 2021, the China Internet Network Information Center (CNNIC) released the 47th Statistical Report on the Development of China's Internet Network in Beijing, showing that “as of December 2020, the scale of China's Internet users reached 989 million, an increase of 85.4 million over March 2020, and the Internet penetration rate reached 70.4%, an increase of 2.5 percentage points over March 2020.” According to the Internet Penetration, more than 50% of the net-citizens are under the age of 40, and among them, the largest number of the net-citizens is students, accounting for 21% as shown in Figure 1. With the increase in the scale of net-citizens and the penetration rate of the Internet, online education has gradually developed. In the context of the Internet era, combined with the needs of the new era for online education, in order to improve the timeliness and effectiveness of online Ideological and political education, it is necessary for online education platforms to explore new ways to innovate the ways and means of online ideological and political education [1].

Ideological and political education is a key link in the fundamental task of online education platforms to improve individual ideological quality, and it is also an important part of online quality education (Figure. 1). With the development of 5G technology, based on the mobile education environment, online ideological and political education has become an important educational path for political education on online ideological platforms in the new era [2]. The new media digital technology represented by the mobile Internet has also brought new challenges to the collaborative management of online ideological and political education platforms while promoting the reform of ideological and political education. Obviously, the construction of a collaborative management mechanism for online ideological and political education platforms in the mobile education environment and the creation of a personalized ideological and political education resource recommendation system have important practical application value for improving the effectiveness of ideological and political education [3].

From February to May 2020, the epidemic caused primary and secondary schools to use the Internet for online teaching. According to the Internet Statistics report, during the epidemic period, many online education application platforms had active users. The number can reach the level of tens of millions. (2) In contrast, in the case of off-campus online education, a number of high-quality teaching platforms have emerged in recent years, many large amounts of financing have been obtained, and the total annual financing has exceeded 10 billion yuan. (3) Online teaching organized by the school during the epidemic period. Classes can only achieve basic functions such as page sharing and audio and video communication, and the off-campus online teaching platform can achieve more diverse functions. On the “bright future” online platform, primary and secondary school principals provide online educational consultation, and their user groups involve more than 200 cities across the country. In addition, the platform also actively develops artificial intelligence technologies such as speech recognition and expression recognition to assist classroom teaching. During the course, real-time interaction, Q&A, classroom detection, voice testing, and other functions can be realized. (1) In addition to the online teaching learning platform, there are also some tools to assist the learning app. For example, Jopshelp is a photo search tool, which can take pictures of the question upload, relying on the text and image recognition function, and present the steps and analysis of the question taken. In addition to taking pictures and searching questions, Homework Help is also autonomous. It has developed functions such as composition search and ancient Chinese search. Because of its convenient function, it is welcomed by many teachers and students, with a total of 800 million users and a monthly average of 170 million users. In addition, there are a series of online teaching in primary and secondary schools such as children's programming and English foreign teachers.

During the new crown pneumonia epidemic, the development of online education has been accelerated, teachers in many schools have adopted the Internet to conduct live teaching, the off-campus online education platform has a variety of teaching forms, and the functional development is relatively mature compared with the in-school teaching. Primary and secondary school students have basically carried out the process of online learning, a certain understanding of online teaching. Besides, the investigation on students' demands for off-campus online education shows that they also expect to provide relevant suggestions for the development of online education.

## 2. The Necessity of Innovating Ideological and Political Education under the Internet Environment

### 2.1. The Need to Grasp the Right to Speak in Ideological Work

Ideology determines the direction of the direction and development of a country's culture, has a bearing on the will of the people, the development of the economy, the stability of society, and the security of the country, and is an extremely important task of our party and our country. With the improvement of mobile network technology, the struggle in the ideological field has become more and more complex [4]. At present, the ideological construction of online education platforms is also facing severe challenges, and the ideological work of online education platforms should take the initiative to open up new positions, learn to use new means, adopt a popular way, firmly grasp the right to speak, and enhance initiative. At the same time, we must also learn to use mobile new media to understand public opinion and grasp the dynamics of their thoughts and behaviors. Under the new mobile media, online education platforms should strengthen the guidance of ideological work, improve timeliness, and enhance the guidance of mainstream awareness to the audience. At present, the Internet is full of some irrational voices and disharmonious discourses, such as the spread of extremely wrong statements such as “Marxism is outdated.” There are also some people who use the guise of so-called “academic research” to distort and slander history in an attempt to impact the mainstream ideology of our country, which must arouse the high vigilance of online education platforms [4].

### 2.2. Practicing the Guidance of Socialist Ideology with Chinese Characteristics

As an online education platform, it must deeply understand the essential characteristics and cultural connotations of socialism and should fully integrate Xi Jinping Thought on Socialism with Chinese Characteristics for a New Era into ideological and political education, especially pay attention to making good use of and giving full play to the Internet, give full play to the advantages of the mobile Internet, and use flexible, diverse, and colorful forms. Do a good job in publicizing and interpreting the socialist ideology with Chinese characteristics, so that, in the world of the audience, it can “see every day,” “every day is new,” and “every day is deep,” strengthen the guidance of the core values of the public, and ensure that the relevant reports of General Secretary Xi Jinping can firmly occupy the headlines of the online education platform. Truly let them sink into their minds and deepen their identification with the theoretical character, practical value, and ideological charm of new ideas [5].

### 2.3. The Internet Has the Characteristics of Respecting and Meeting the Individual Needs of Online Education Audiences

According to the previous survey, compared with the traditional Internet, the mobile Internet has the advantages of learning and information communication anytime and anywhere and can fully use the audience's “fragmented time” to improve learning efficiency, which provides convenience for the public to pursue values such as autonomy and individuality [6]. First, the mobile Internet provides the audience with the function of independent choice. The audience's sense of autonomous choice is strengthening, their thinking is becoming more personalized, they like to act in their own way, using the Internet to express themselves, and the mobile Internet provides them with richer, more humane content and flexible operating methods, which can help them achieve this autonomous need [7]. Second, the mobile Internet provides personalized choice needs for the audience. Audiences have a strong desire for differentiation and personality, and it caters to their choices in a flexible way. Third, the mobile Internet provides practical functions for students' learning and life. The mobile Internet can provide a variety of practical information and services for the audience and can meet the needs of different levels of knowledge. Fourth, the mobile Internet provides the possibility for ideological and political education to promote online education. The development of Internet technology has realized the technology of big data extraction, called cloud computing. Under the support of cloud technology, users have realized “ubiquitous learning,” that is, users can learn under any location, time, and equipment conditions, and they do not need to maintain equipment and software, learning resources are enriched, learning costs are reduced, and convenience is enhanced [8].

When schools effectively combine ideological and political education with Internet information technology, they can change the status quo of single teaching forms and boring teaching content to a certain extent. By using the Internet information technology, students' interest in independent learning is increased, making students consult materials anytime and anywhere while actively thinking. It is conducive to cultivate students good habits and master good methods in learning. For example, in recent years, schools have actively created red websites for campus ideological and political education, which are diverse in form and rich in content, which increase the interest of students' learning and improve our personal cultivation.

## 3. The Connotation of Online Ideological and Political Education

### 3.1. Characteristics of Online Ideological and Political Education on Online Education Platforms

Network ideological and political education is a form of ideological and political education with college students as the main body of education [9], in accordance with the teaching plan and ideological and political education theory of the online education platform, give full play to the role of Internet technology, and realize the online education platform objectives of ideological and political education [10]. The educational means of network ideological and political education have their own characteristics: first, openness—the Internet system has no boundaries of regional space, and network information can be spread to any place in the world in a relatively short period of time, with super influence and penetration. The second is timeliness—the Internet is the world's fastest information highway, and its information update and dissemination speed is unmatched by traditional media. The third is equality—network ideological and political education is more flexible than the traditional way and reflects the characteristics of equality in the relationship between educators and the subjects of education [11]. The fourth is interactivity, and there is an activity process of equal communication and effective interaction between educators and educational objects, which has obvious interactive characteristics [12].

### 3.2. The Development Trend of Online Ideological and Political Education on Online Education Platforms

Network ideological and political education is a new form of education in ideological and political education, and its development trend is mainly reflected in the following aspects: the coverage penetration function is stronger, and the coverage penetration function refers to the ideological and political education information provided by the educated through the network of accessing the carrier of ideological and conceptual transmission, so that it is affected and influenced [13]. Traditional means of ideological and political education are often subject to factors such as venue and time, the coverage of education is relatively limited, the development of the network can make ideological and political education break through the limitations of time and space, through one-to-many and many-to-many network ideological and political work platforms, to help promote the whole staff, the whole process, and all-round education [14]. Second, it is more innovative. As an innovative carrier of ideological and political education, the Internet is an inevitable requirement for today's social development and the development of ideological and political education. Network political education can adapt to the diversified and convenient needs of young students' access to information channels, guide users to join the interactive activity process, allow teachers and students to exchange opinions on an equal footing, change the mode of communication between teachers and students, and make the breadth and depth of communication reach a new level [15]. In addition, online ideological and political education is more oriented, making the Internet a new front for ideological and political education, passing on the core socialist values to students, strengthening their ideals and beliefs, and guiding young students to continuously improve their ideological level, political awareness, moral character and cultural literacy. Great virtue, public morality, and strict private morality can make users to become qualified socialist builders and successors, leading to all-round development of morality, physical fitness, beauty, and labor [16] as shown in Figure 2.

The rapid development of the modern Internet information technology, with its large amount of information and wide coverage, has not only become the main means and way for students to seek knowledge but also further expanded the cultural and entertainment life of college students. For example, with the help of the Internet, worldwide exchanges and interactions can be learned about real-time information at home and abroad without leaving home; find friends with the same interest on the Internet, encourage each other, and move forward side by side. Increase common topics with others, expand the scope of interpersonal communication, and increase social participation. All these help college students to open their minds, so that they have the ability to respond flexibly to problems, learn from each other, and gradually adapt to society.

## 4. The Challenges Faced by Online Education Platform Ideological and Political Education in the Network Environment

### 4.1. The Impact of Heterogeneous Nonmainstream Values

The Internet has produced a huge penetration and impact on social life, and the proportion of student users in the total number of net-citizens is not low [17]. First, cybersecurity issues are frequent. In terms of network security issues, online fraud and personal information leakage are emerging in an endless stream, and there are more student victims in telecommunications fraud cases. Second, cyberspace is open and inclusive. In cyberspace, pluralistic values can be easily disseminated, and all kinds of heterogeneous nonmainstream values are more likely to have an impact on college students [18]. However, college students have not yet formed correct ideological values and lack the ability to correctly distinguish multiple values in cyberspace, which is prone to misconceptions [19].

The information content on the Internet is complex, and the speed of dissemination is very fast. Some websites operate in violation of the law, and even there are illegal acts that make the viewer passively accept pornographic information, so students are easily addicted to it while the convenience brought by network habits, and some students are difficult to resist its attractiveness, resulting in declining academic performance or even more serious consequences. Not only this, Internet addiction will also reduce students' normal life time such as thinking, sleeping, and communicating, affecting students' vision, hearing, memory, and reaction ability, causing both physical and psychological damage. It is easy to lose the real self because of the long-term indulgence in online space, it is easy to confuse the virtual online character with the real character, and in the long run, it becomes a “communication idiot.” However, if the negative behaviors and psychology exposed in the network are transmitted to users, it is not conducive to a healthy campus atmosphere, and even affect academic and physical and mental health.

### 4.2. Traditional Ideological and Political Teaching Classrooms Lose Their Attractiveness to Students

With the popularization of smart phones and the Internet, teachers and students are gradually equal in accessing information, teachers no longer have the priority of obtaining knowledge, and students can freely swim in the ocean of online information and directly obtain information and communicate. Therefore, the Internet age has changed the relationship between teachers and students to “give” and “receive,” making a single traditional ideological and political teaching classroom unattractive to students, teachers need to improve their network skills, be good at using diverse network information resources, and create a rich and colorful teaching classroom [20].

The continuous expansion of the massive information in the Internet era makes it more difficult for the huge user groups to screen the massive information resources. With the continuous accumulation of massive information every day, users find the desired information in it is simply to find a needle in a haystack and, at the same time, accompanied by the burial of high-quality resources, resulting in a great waste of resources. Personalized recommendation department is an effective technical means to help users quickly identify and screen out useful information for users and help high-quality resources to users who need it. Personalized recommendation system is generally composed of three important modules (Figure 3). First, the user interest model is generated after the analysis of users' personal behavior data record and, second, the establishment of the recommendation project model, and the recommendation engine of end user interest model and recommendation project model.

Target users and similar demand users recommend their video resources of interest. That is, the core point is to take the similarity of users and obtain similar users through the relevant characteristics of users. Then, similar users speculate the interest of their target users and then combine other influencing factors to generate the recommendation list. For its implementation, there are usually three steps (Figure 4):

### 4.3. A Single Communication Method Cannot Achieve the Goal of Educating People

The online education platform ideological and political education carries an important function of educating people, which is related to the question of “for whom to cultivate people, what people to cultivate and how to cultivate people” [12]. Timely acquisition and grasp of students' ideological dynamics is an essential part of education and teaching, which requires good communication and exchange between teachers and students. In the Internet era, the way of communication and communication is increasingly diversified, the face-to-face teaching method of online education platform ideological and political education still occupies the main position, and students only passively accept theoretical knowledge. In the network environment, college students have developed a variety of learning needs and personalized learning habits, relying only on a single top-down communication method, unable to perceive the true thoughts of students, and teachers cannot know the changes in students' ideas and concepts.

### 4.4. Solidified Teaching Content Cannot Meet the Needs of Students

The content of traditional ideological and political education is mainly based on the textbooks of ideological and political science, mainly including Marxist philosophy, the theory of socialism with Chinese characteristics, the outline of modern Chinese history, the cultivation of ideological character, and current affairs and politics. At the same time, the overall planning and outline selection of ideological and political education also occupy part of the content. However, in the network environment, college students receive information in more diverse ways, and can feel social hot information faster and more. At this time, teachers and textbooks are no longer the main sources for students to receive relevant theoretical knowledge. If the ideological and political education of the online education platform is still based on fixed textbook content to provide ideological education, it can not meet the knowledge needs of students, nor can it adapt to the habits of students to obtain information, and it will also affect the teaching effect.

### 4.5. Excessive Use Leads to Students' Gradual Loss of Social Skills

The use of the Internet to communicate has become a common phenomenon around the world, and people use it for work, entertainment, dating, etc. The Internet can break through the limitations of time and space and weaken the traditional way of communication, people can easily make friends of different personalities through the Internet, from getting emotional and self-worth satisfaction. However, when college students are addicted to online communication, they will inevitably ignore the interaction with others in real life, and over time, they will be estranged from their classmates, teachers, and parents, and there will be a strong psychological gap, which will gradually reduce their social communication skills in real life, resulting in lack of self-confidence, avoidance psychology, and gradually interpersonal barriers.

## 5. The Network Environment Brings Opportunities for Ideological and Political Education on Online Education Platforms

With the help of Internet information technology, massive information resources can further enrich educational resources, information teaching platforms can also be effectively built, coupled with the diversification trend of education subjects and the strengthening of education pertinence, and online education platform ideological and political education can achieve a higher level of development and show a stronger educational effect.

First, create a main classroom for ideological and political education. Through the arrangement of collective teaching, individual counseling, individual Q&A and section testing, the traditional ideological and political classroom teaching methods are transformed, and the ideological and political teaching and the Internet are highly integrated, so that the classroom teaching content is more advanced and interesting, and the learning methods are more modern. The audio, film, and television materials that students are interested in are introduced into the study of ideological and political theory class. The class is simple and easy to understand so that students can more easily analyze and solve difficult problems in real life.

Second, use the Internet platform to promote auxiliary functions. Through the combination of multiple online platforms, students are provided with a variety of learning channels. Teachers actively open online tutoring services, enter students' learning circles and social circles through QQ, WeChat, mailbox, Weibo and other forms after class, cultivate and practice modern teacher-student relationships, and always solve problems in life and learning for students. At any time, we should grasp the ideological dynamics of students, minimize the negative impact of the Internet, and enable each student to have a solid grasp of the content of ideological and political education in colleges and universities, taking students as top concern.

### 5.1. Massive Information Provides Rich Resources for Teaching Ideological Politics

In view of the diversification of information and the efficiency of technology in the network environment, the online education platform Sizheng Education can obtain rich teaching resources from it [14]. On the one hand, the rich and diverse information resources in the online environment can become the material for ideological and political education on the online education platform. In cyberspace, a variety of ideological values and social information are widely disseminated, among which information resources that conform to the core values of socialism are compatible with the knowledge of ideological and political theory can become the materials for ideological and political education on the online education platform. Network technology, on the other hand, updates educational resources in real time. Using the Internet information technology in the network environment, teachers can realize the overall macro control of the development of contemporary college students and current ideological and political education, realize the timely update of teaching resources, and ensure the timeliness of educational content.

The online learning platform guides users to complete the preclass learning evaluation tasks with good credibility and analyzes the users' learning style. Furthermore, the system recommends the corresponding learning resources according to the user's learning style (as shown in Table 1).

### 5.2. Promoting the Construction of Educational Resource Libraries and Information-Based Teaching Platforms

On the one hand, educators can build a library of educational resources. On the basis of obtaining many educational information resources, online education platform ideological and political educators can build a political education resource library, effectively sort out and analyze teaching resources with big data, cloud computing, and other technologies, and store them in the resource library to provide resource references and educational examples for educators across the country. On the other hand, the network environment can also bring an information-based teaching platform and innovative forms of education to education. The open network information environment can help ideological and political education break through the traditional time and space restrictions, build an information-based teaching platform, put ideological and political education on the network platform, provide educators and students with online teaching and communication channels, and also promote the innovation of educational forms.

In the process of school learning, students mainly learn through the guidance of the teacher, and sometimes through the form of self-study, because students' enthusiasm for learning, learning basis, learning talent and other factors are different, they will develop different learning ability. And with the continuous improvement of students' learning period, they will learn more and more difficult knowledge, and the corresponding students' learning level will continue to improve. Students have different learning resources, and different students in the same grade also have different learning abilities. Students with strong learning ability are generally able to and are willing to learn resources that are more difficult, while students with weak learning ability can only learn less difficult resources. Therefore, students' learning ability should be considered in the student model. This paper uses the survey questionnaire to determine the value of students' learning ability. In conclusion, we can summarize the student model in Table 2.

### 5.3. Promoting the Diversified Reform of Educational Subjects

Under the background of the Internet information technology, many entities related to ideological and political education can participate in education, realize the synergistic linkage with educators on the online education platform, open timely interactive exchanges with the help of cyberspace, and help the online education platform ideological and political education to achieve diversified development. In the network environment, all kinds of ideological and political education entities can jointly carry out educational work, provide educators with diversified educational materials and forms of education, and also help educators better understand the learning and life characteristics of contemporary college students and enhance the affinity and pertinence of education.

### 5.4. Enhancing the Pertinence of Education

With the student user model, the educational resource model and the matching formula, we can establish the whole educational resource personalized recommendation scheme.  Figure 5 describes the overall process of the educational resource personalized recommendation scheme in this paper.

Big data technology based on analysis has created more possibilities for prediction, and the wide application of this prediction in the field of ideological and political education on online education platforms will inevitably improve the effectiveness of education. Under the influence of the network environment, college students actively participate in information acquisition or hot discussion, more autonomous and personalized; in view of this, online education platforms think about politics and education. Education needs to use big data, cloud computing, and other information technologies to increase the collection and analysis of college students' learning data, effectively grasp the thinking characteristics and ideological dynamics of college students on the basis of ensuring security and privacy, and, on this basis, select educational content and education methods in a targeted manner, so as to better meet the characteristics and needs of college students and then achieve efficient development of education.

## 6. The Construction of a Management Mechanism for Ideological and Political Education Platforms in the Network Environment

### 6.1. Construction of Guidance Mechanisms

The guidance mechanism of the network ideological education platform refers to the gradual formation of an institutionalized mode of operation through the interaction and integration of educational resources in the process of teaching students to continuously improve their ideological level, political awareness, moral character, and cultural literacy and in the process of achieving great morality, public morality, and strict private morality. Proceeding from adhering to the socialist direction of running schools and the fundamental task of cultivating people with moral integrity, we should grasp the ideological context of students, make them accept the guidance of the network ideological and political education platform, cultivate students' patriotic feelings, sense of social responsibility, innovative spirit, and practical ability, and realize the all-round development of students' morality, intellectual, physical, and aesthetic work. Due to the complexity of the mobile network technology, it poses greater challenges to ideological and political teachers, requiring ideological and political teachers to master advanced information processing technology, learn to effectively screen relevant knowledge, and flexibly apply it to the actual daily ideological and political curriculum education and teaching. In the new era, ideological and political teachers must have a variety of teaching capabilities, make full use of their own teaching knowledge and skills to guide students to selectively absorb relevant information, and learn to use the knowledge and information in the mobile network to effectively study political thinking, and for the problems and teaching knowledge difficulties in learning, they can use Weibo and WeChat to achieve interactive communication with teachers. Teachers can also grasp the learning situation of students in real time, make comments, or carry out targeted education guidance to improve the effectiveness of ideological and political education.

### 6.2. The Construction of a Sharing Mechanism

The integration of online ideological and political education resources means that various teaching resource modules should be integrated and adjusted with each other, solve the problem of mutual cooperation between various courses and ideological and political courses, form a synergistic effect, and complete the goals of ideological and political education. The construction of the sharing mechanism reflects the educational function, which enables the platform to continuously improve the work system, teaching system, and content system of curriculum ideology around the goal of talent training. Through the integration of goals, functions, and information, we will dig deep into the ideological and political education resources contained in the curriculum and teaching methods and gradually build a curriculum ideological and political teaching resource system with rich types, progressive levels, and mutual support. Schools should actively adapt to the trend requirements of new media integration, use the decentralized distributed storage and consensus mechanism of block-chain technology, break down platform barriers, and integrate and share scarce and high-quality teaching resources. Teachers can use social media such as Weibo, WeChat, and public accounts and can also use short video community platforms such as Douyin, Kuaishou, and Station B to achieve interactive exchanges between teachers and students and facilitate fierce discussions on ideological and political issues in the classroom. Teachers can also publish some topics or hot topics and news events related to the development of the national situation, give some pertinent opinions or suggestions that are in line with the core values of socialism and world outlook, guide students to participate in discussions, and help students establish a correct world outlook and outlook on life.

For the evaluation of the recommendation results, the user evaluation will start from three perspectives—whether it meets the learning objectives, the learning interest, and the recommendation results and analyze the utility of the recommendation results of different algorithms (the evaluation results), as shown in Table 3. The final ratio in the table is the proportion of the number of users positive. The objective and subjective results show that students have high satisfaction with the improved algorithm, indicating that the degree of personality of the recommended results of the improved algorithm is improved.

### 6.3. Establishment of Safeguard Mechanisms

The guarantee mechanism of the online ideological and political education platform is based on the objective needs of education and teaching, through organizational management, process management, and safety management, adhering to the unity of theory and practice, combining the offline ideological and political education small classroom with the online ideological and political education classroom and achieving the expected goals of ideological and political education. Once the platform management mechanism is formed, it will spontaneously and dynamically guide and decide on management behaviors according to certain laws and orders to achieve effective management:

1. Organizational guarantee: organizational management refers to the establishment of the organizational structure of the platform through design, the rational allocation of personnel, the formulation of rules and regulations, the clarification of the relationship of responsibility and authority, the provision of the necessary organizational carrier and organizational support for the operation of the platform, the development of management of educators and the educated, the coordination of the relationship between the two, and the provision of organizational guarantee for the better realization of the goals of ideological education [19]. The relevant functional departments of the school may formulate rules and regulations for online ideological and political education, clarify management responsibilities, coordinate the division of labor in management, coordinate the allocation of personnel, and exert the cohesion of all levels of organizational structures to form a management synergy.
2. Process management: process management refers to the use of a practical approach to planning, controlling, and improving the effectiveness, efficiency, and adaptability of processes. Institutionalized process management contributes to the smooth operation of the network platform. In order to make the platform operate effectively, the process method should be used to identify the process of interrelation and role between the management responsibility, guarantee responsibility, coordination responsibility, and incentive means of the platform, and implement continuous control and continuous improvement of the connection, combination, and interaction between them, so as to improve the operational efficiency of the network ideological education platform and enhance the satisfaction of the use of the platform.
3. Safety management: safety management refers to the main use of modern safety management principles, methods and means, analysis, and study of various unsafe factors, from the technical, organizational, and management to take effective measures to solve and eliminate unsafe factors, to prevent accidents. The network security management system that conforms to the law of network development is the institutional guarantee for colleges and universities to have a safe and stable network media environment, and scientific and effective system design can ensure the healthy and orderly development of the campus network of colleges and universities. With the development of the Internet, new media such as Weibo, WeChat, APP clients, and short video platforms are increasingly involved in the operation of new media platforms in colleges and universities, and the intervention of social forces provides a fast and convenient network interaction platform for ideological and political education, while also bringing pressure to the network security management and public opinion monitoring of colleges and universities, requiring colleges and universities to further improve the construction of security systems, so that a sound network security management system can escort colleges and universities in network ideological and political education.

### 6.4. The Construction of Assessment Mechanisms

The evaluation of the online ideological and political education platform is based on the objectives and requirements of ideological and political education, on the basis of systematically and scientifically sorting out and analyzing relevant information on ideological and political education and using certain evaluation indicators and methods to measure and evaluate the elements, processes, and effects of ideological and political education. Through teachers, students, content, carriers and environment, and other elements, a comprehensive evaluation of the online ideological and political education platform of colleges and universities is carried out, and its performance, quality, and operational status are evaluated. It is necessary to think whether the educational elements are complete and high quality, whether the comprehensive application of various elements is effective, whether the education program is keep pace in time and real, and whether the system is perfect. It is also necessary to look at the organizational situation of each stage and link in the process of implementing ideological and political education, the transition and articulation between each other, and whether the relationship between subject and object can be correctly handled well in the teaching process and the combination of the leading role of teachers and the main role of students. Furthermore, it is more necessary to examine the actual effects of ideological and political education, which are mainly reflected in the development and changes of students' thinking and behavior. The establishment of the evaluation mechanism of the online ideological and political education platform provides an important basis for strengthening and improving ideological and political work and evaluating the effectiveness of ideological and political education, and its purpose is consistent with the goal of ideological and political education, and in essence, it is to make value judgments on the social and individual effects of ideological and political education [20].

### 6.5. Construction of Teacher Training Mechanism

Under the background of the new era, ideological and political workers should continuously improve their political quality and network literacy, accurately grasp the convergence point between ideological and political education and information technology, skillfully apply information technology to build a smart teaching platform, and firmly grasp the leading role of online ideological and political education. General Secretary Xi Jinping stressed at the 2019 School Ideological and Political Theory Teachers' Forum that the ideological and political curriculum is a key course for implementing the fundamental task of Lide Shuren, the role of the ideological and political class is irreplaceable, and the teacher team of the ideological and political class has a heavy responsibility. The “Opinions on Strengthening and Improving the Ideological and Political Work in Colleges and Universities under the New Situation” also pointed out: it is necessary to strengthen the construction of the contingent of teachers and special forces. The ideological and political work contingent and the party affairs work contingent of colleges and universities have the dual identities of teachers and managers and should be included in the overall plan for the construction of the contingent of qualified personnel in colleges and universities, forming a work force that is mainly full-time, combines full-time and part-time work, has sufficient quantity, and has excellent quality. “To improve the training mechanism of the network ideological and political education team, it is necessary to establish a perfect talent guarantee system for the ideological and political teacher team in light of their own actual conditions, study and issue a series of supporting documents and policy measures, and build a high-quality ideological and political work team that combines specialization and combination.” It is also necessary to organize education and training, strengthen the practical training of the ideological and political work contingent, improve the incentive mechanism, and promote the professionalization and professionalization of the ideological and political work contingent.

## 7. Conclusion

All in all, combining the ideological and political education of college students with the advanced and convenient Internet is one of the important ways which brought China from lagging behind to being the first in education. The networking of education has become the trend of the trend, the boundaries of users are also expanding, and colleges and universities should actively pay attention to the changes in the political ideology of college students and the health of the network environment when carrying out ideological and political education for students. Opening up new learning channels for students will help improve the degree of enthusiasm of college students in ideological and political study and can also promote the comprehensive development of contemporary college students.

As the main force in the new era, when the country is becoming more and more open, science and technology are becoming more and more powerful, and the culture is becoming more and more abundant, we must resolutely adhere to the bottom line of our own thinking, choose to accept positive and beneficial culture and information, in order not to lose ourselves in this complicated Internet+ era and to truly add our own strength to this rapidly developing country and society. As a high-quality talent of the country, it is necessary to have good political thinking, establish a correct world outlook, outlook on life, and values, use a wide range of network resources to open up thinking, enrich themselves, and lay a good foundation for entering society in the future. At the same time, ideological and political education in colleges and universities should also keep pace with the times, actively respond to all the adverse effects and consequences brought about by the Internet, and comprehensively grasp the correct use of the Internet by college students through political theory, case publicity, and regular supervision, so as to avoid the negative impact of excessive consumption of the Internet and promote the vigorous development of college students.

## Figures and Tables

**Figure 1:** Scale of net citizens and Internet penetration rate.

**Figure 2:** Market size of the online education industry.

**Figure 3:** The recommended model.

**Figure 4:** A user-based recommendation system.

**Figure 5:** Overall flow chart of the personalized recommendation program for educational resources.

**Table 1:** Explicit classification of learning styles.

Style dimension	Dimension classification	Features	Relevant recommendations
Information processing	Active type	They prefer to verify ideas through experiments, do first and then think, and prefer discussion and teamwork	For example, discussion area and forum
	Contemplative type	They prefer to learn new things through thinking, think first and then do, and prefer to think and work independently	For example, blog and log

Information perception	Perceptual type	More inclined to examples and memories	More specific examples, such as algorithm application
	Intuitive type	More abstract and deductive	More abstract derivation, such as algorithm extension

Information input	Speech type	Prefer explanatory text	PPT, literature
	Visual type	Prefer pictures, videos, etc.	Video and mind map

Information understanding	Comprehensive type	General understanding first and then in-depth	More courses or knowledge navigation marked by “previous and next sections”
	Sequence type	Learn step by step	More general outline

**Table 2:** The student model.

Category	Project	
Demographic characteristics relatedto learning background	Gender	
	School	
	Academic section	
	Subject	
	Major	

Characteristics related to learning style	Physiological dimension	Visual type
		Auditory type
		Kinesthetic type
	Cognitive dimension	Field independent type
		Field dependent type

Characteristics related to learning ability	Learning ability	Very strong
		Strong
		Poor
		Very poor

**Table 3:** Satisfaction analysis.

Recommendation algorithm	Learning objectives (%)	Learning interest (%)	Recommendation result satisfaction (%)
Traditional collaborative filtering algorithm	58.5	68.5	73
Improved collaborative filtering algorithm	70.5	78.5	93

## Data Availability

The labeled data set used to support the findings of this study is available from the corresponding author upon request.

## References

[1] Fan G., Meng F. Personalized recommendation algorithm for curriculum-and politics-oriented hybrid teaching resources.

[2] Yang F. (2020). Analysis on the relationship between the media literacy of film & television and the innovation of ideological and political education of contemporary college students. *Lifelong Education*.

[3] Gao Y. The connotation and function mechanism of ideological and political education of big data.

[4] Bhutoria A. (2022). Personalized education and artificial intelligence in USA, China, and India: a systematic review using a human-in-the-loop model. *Computers and Education: Artificial Intelligence*.

[5] Zhao C. (2020). Characteristics and changes of audience psychology in ideological and political education. *Revista Argentina de Clinica Psicologica*.

[6] Han W. (2020). Using information technology to improve ideological and political education and student management efficiency in colleges. *Journal of Physics: Conference Series*.

[7] He L. (2021). Innovation strategy of network ideological and political education based on big data. *Journal of Physics: Conference Series*.

[8] Yang Y. (2021). On the normalization path of online teaching of ideological and political course in colleges and universities in the “post epidemic” era. *Journal of Contemporary Educational Research*.

[9] Pianzola J., Trechsel A. H., Vassil K., Schwerdt G., Alvarez R. M. (2019). The impact of personalized information on vote intention: evidence from a randomized field experiment. *The Journal of Politics*.

[10] Lv Z., Chen J. (2022). Research on big data administration promotion strategy of ideological and political construction in institutions of higher learning from the perspective of cognitive psychological study. *Forest Chemicals Review*.

[11] Li L. (2019). *Innovation Path on Ideological and Political Education in Colleges and Universities in the New Media Era*.

[12] Peng P., Fu W. (2022). A pattern recognition method of personalized adaptive learning in online education. *Mobile Networks and Applications*.

[13] Zhang L. (2018). The relationship between self-efficacy and job burnout of ideological and political teacher based on quantitative and qualitative analysis. *Neuroquantology*.

[14] Lu D. (2018). Based teaching model of ideological and political course under computer network environment. *Educational Sciences: Theory and Practice*.

[15] Du W. Design and application of learning APP for ideological and political course based on android & SSH.

[16] Le H., Maragh R., Ekdale B., High A., Havens T., Shafiq Z. Measuring political personalization of google news search.

[17] Regan P. M., Steeves V. (2019). Education, privacy, and big data algorithms: taking the persons out of personalized learning. *First Monday*.

[18] Hwangbo H., Kim Y. S., Cha K. J. (2018). Recommendation system development for fashion retail e-commerce. *Electronic Commerce Research and Applications*.

[19] Saito T., Watanobe Y. (2020). Learning path recommendation system for programming education based on neural networks. *International Journal of Distance Education Technologies*.

[20] Rana A., Deeba K. (2019). Online book recommendation system using collaborative filtering (with jaccard similarity). *Journal of Physics: Conference Series*.

